The article "Biomechanical Analysis of Different Internal Fixation Combined with Different Bone Grafting for Unstable Thoracolumbar Fractures in the Elderly" was retracted in 2024. Reasons: signs of a paper mill; suspected computer-generated content; unreliable results or conclusions; concerns about the data.

# Biomechanical Analysis of Different Internal Fixation Combined with Different Bone Grafting for Unstable Thoracolumbar Fractures in the Elderly

**DOI:** 10.1155/2022/2863379

**Published:** 2022-04-25

**Authors:** Qisong Shang, Yuqing Jiang, Wenhui Sheng, Pengyuan Han, Junru Zheng, Xing Wang, Bing Wu

**Affiliations:** ^1^Department of Spinal Surgery, The Third Affiliated Hospital of Shihezi University Medical College, Shihezi, 832000 Xinjiang Uygur Autonomous Region, China; ^2^Department of Spinal Surgery, Changzhou Second People's Hospital Affiliated to Nanjing Medical University, Changzhou, 213000 Jiangsu Province, China

## Abstract

This research was developed to accurately evaluate the unstable fractures of thoracolumbar before and after surgery and discuss the treatment timing and methods. Three-dimensional (3D) finite element method was adopted to construct the T_12_-L_5_ segment model of human body. The efficiency of percutaneous kyphoplasty (PKP) and percutaneous vertebroplasty (PVP), two commonly used internal fixation procedures, was retrospectively compared. A total of 150 patients with chest fracture who received PKP or PVP surgery in our hospital, and 104 patients with the same symptoms who received conservative treatment were collected and randomly rolled into PVP group (75 cases), PKP group (75 cases), and control group (104 cases). Visual analog scale (VAS) score and Oswestry disability index (ODI) of patients were collected before and after surgery and 2, 12, and 24 months after surgery. Then, the anterior and central height of the patient's cone and the kyphosis angle were calculated by X-ray. Lumbar minimally invasive fusion system and lumbar pedicle screw rod system were established by computer-aided design (CAD), and the biomechanical characteristics were analyzed. The results showed that there was no substantial difference in VAS score and ODI score between PKP and PVP (*P* > 0.05), but they were higher than those of the control group (*P* < 0.05). The anterior edge and middle height of vertebra in the two groups were higher than those in control group (*P* < 0.05), and the increase in PKP group was more substantial (*P* < 0.05). The kyphosis of the two groups was smaller than that of the control group (*P* < 0.05), and the decrease of the kyphosis of the PKP group was more substantial (*P* < 0.05). In summary, the thoracolumbar segment model established by 3D finite element method was an effective model, and it was verified on patients that both PKP and PVP could achieve relatively satisfactory efficacy. The implantation of the new internal fixation system had no obvious effect on the lumbar movement. This work provided a novel idea and method for the treatment of senile thoracolumbar unstable fracture, as well as experimental data of biomechanics for the operation of senile unstable fracture.

## 1. Introduction

China has entered the aging society since 2002. According to relevant data estimation, there are 44.49 million patients with osteoporotic vertebral compressive fracture (OVCF) in China at present, with a high growth rate of 1.81 million cases per year. For which, the social medical expenditure is as high as 9.45 billion yuan [1]. According to the corresponding model study, by 2020, the number of new OVFC patients over 50 years old will reach 1.49 million [2]. For OVCF, more than 45% of spinal injuries occurred between lumbar T_11_-L_1_ [3]. Unstable fracture of thoracolumbar refers to thoracolumbar fractures, which are prone to displacement or re-displacement after reduction, accounting for half of thoracolumbar fractures. Unstable fracture is an important culprit of anatomical structure injury and deformity. Of which, 20-40% of thoracolumbar fractures are associated with nerve injury, which will lead to persistent nerve function impairment and even paralysis in patients [4–6].

As a common spinal disease in elderly patients, spinal fracture is often associated with osteoporosis. Elderly patients with spinal fracture and long-term bed rest will not only cause a variety of diseases or even death, but also bring numerous burdens to the family and society [7]. Therefore, the treatment of acute symptomatic osteoporotic thoracolumbar compression fracture patients is imperative for the prevention of osteoporosis in the general healthy elderly. Helping patients get out of bed as soon as possible and become independent is the primary goal of osteoporosis research. At present, percutaneous vertebroplasty (PVP) and percutaneous kyphoplasty (PKP) are the mainstream surgical methods for the clinical treatment of elderly thoracolumbar unstable fractures [8], whose efficacy has been fully affirmed by spine surgeons [9]. Although there are many trials comparing the efficacy of PVP and PKP, and the two vertebral amplification methods have their advantages and disadvantages, the choice of the two surgical methods is still partly controversial [10].

In terms of spinal internal fixation for osteoporosis patients, China published in 2019 *Chinese Expert Consensus on Spinal Internal Fixation for Elderly Osteoporosis* and *Clinical Guidelines for Vertebrae Enhancement for Acute Symptomatic Osteoporotic Thoracolumbar Compression Fractures*. In the *Clinical Guidelines for Vertebrae Enhancement for Acute Symptomatic Osteoporotic Thoracolumbar Compression Fractures*, PVP is recommended at level I for acute symptomatic OVCF, and PKP is recommended at level II. However, if the injured vertebra height needs to be restored, PKP (level I recommendation) is performed [11, 12].

However, the bone density of elderly patients is different from that of ordinary young and middle-aged patients. They have low bone density and poor physical quality, and some of them are accompanied by other diseases of aging. Therefore, the choice of appropriate internal fixation system and effective surgical method plays a decisive role in the solution of internal fixation failure in elderly patients. According to the clinical follow-up of elderly patients with thoracolumbar instability fracture after surgery, most of them will develop new vertebral fractures after surgery, which are often located near the cone at the treatment site. Therefore, the pyramidal biomechanical data analysis and its performance evaluation in elderly patients with fractures are the primary issues to be addressed [13, 14].

Finite element analysis is an emerging biomechanical research method, which divides the target structure that is difficult to analyze into a finite number of unit aggregates, and it is used to accurately simulate the structure of the spine and internal fixation. By applying different loads, the biomechanical responses of the spine and internal fixation were obtained qualitatively and quantitatively, and targeted prevention methods were proposed to guide the surgical design [15–18].

At first, electrical measurement and photoelastic methods were used to study the spine. However, these methods were limited by the anatomical structure of the spine and the complexity of various material parameters and stress distribution, so it was often difficult to obtain the overall dynamic information. With the emergence of finite element analysis, all the relevant data of the spine can be reflected in mathematical form, and the internal stress and strain of the structure can be reflected as much as possible. By changing any parameter, the change information of the whole structure can be obtained, which is the most important advantage of finite element analysis.

In summary, the 3D finite element model of human cone was established to simulate the force of thoracolumbar vertebra and analyze the stress distribution of spinal functional units. The biomechanics of thoracolumbar fracture and internal fixation were studied. A total of 150 patients treated by convex plasty and 104 patients treated conservatively at the same time in our hospital were selected as the research objects, among which 75 patients in the surgery group were treated with PKP and 75 patients in the surgery group were treated with PVP. The control group was treated with conservative therapy. Follow-up was conducted before and after treatment and at 2, 12, and 24 months. Visual analog scale (VAS), Oswestry disability index (ODI), and X-ray were employed to calculate the changes of the anterior and central height of the cone, as well as the kyphosis angle of the patients to evaluate the therapeutic effect of the two surgeries. Moreover, the finite element models of lumbar minimally invasive fusion system and lumbar pedicle screw rod system were established by using CAD technology to conduct quantitative biomechanical evaluation and accurate repair of early thoracolumbar fracture.

## 2. Materials and Methods

### 2.1. Research Objects

A total of 150 patients treated with vertebroplasty in our hospital and 104 patients of the same type treated with conservative treatment were recruited as the study subjects. Of the 150 vertebroplasty patients, 75 patients in the surgery group were treated with PKP, and 75 patients in the surgery group were treated with PVP.

Inclusion criteria are as follows: (i) the patient was identified with osteoporotic vertebral fracture; (ii) the patient had indications for surgery; (iii) the bone mineral density of the patient was less than or equal to -2.5; and (iv) patients with conservative treatment that cannot achieve better efficacy.

Exclusion criteria are as follows: (i) patients with malignant or metastatic tumor in the cone; (ii) the patient had chronic disease and cannot receive surgery; (iii) the patient also had hemorrhagic disease; (iv) patients with neurological symptoms or spinal canal accounted for more than one-third; and (v) the patient had local systemic or spinal infection.

There were 75 patients in PVP group, including 12 males and 63 females, aged 52-89 (67.42 ± 8.62) years. Fracture cone distributions were T_12_ of 32 cases, L_1_ of 29 cases, and L_2_ of 14 cases.

There were 75 patients in the PKP group, including 17 males and 58 females, ranging from 54 to 86 (65.28 ± 9.71) years old. Fracture cone distributions were T_12_ of 29 cases, L_1_ of 36 cases, and L_2_ of 10 cases.

A total of 104 patients in the control group received conservative treatment, including 20 males and 84 females, aged 51~88 (66.36 ± 10.32) years. As for the fracture cone distributions, there were 46 cases of T_12_, 39 cases of L_1_, and 19 cases of L_2_.

Before and after treatment, X-ray images were used to calculate the height of the anterior and central cone, and the kyphosis angle of patients in the two groups, and the data were compared. Follow-up was conducted at 2, 12, and 24 months. VAS and ODI were used to evaluate the treatment effect of the two groups.

The clinical data of the two groups were comparable.

### 2.2. Complete Spine T_12_-L_5_ Section Data Acquisition

Siemens SENSATION 16-slice multi-spiral CT was employed to perform continuous parallel scans of the spine of a healthy male volunteer. The generated cross-sectional file was imported into the MIMICS 10.0 of Materlise, Belgium. Threshold was set as 226-2,976. The parts that did not conform to the selection of T_12_-L_5_ vertebrae were removed, and the missing gaps were filled. A 3D model was generated, and mesh smoothing was performed.

### 2.3. Computer-Aided Design (CAD) Post-Processing

The data was imported into ANSYS12.0 for preprocessing to generate 3D volume. Then, the 3D body was imported into the CAD software SolidWoeks2010. The generated model was processed in detail, and the cone was polished, filled, and assembled. Finally, a complete 3D model was established.

### 2.4. Finite Element Model Establishment

The model was imported into ANSYS Workbeach for finite element analysis preprocessing. Material parameters of the model were mainly selected according to literature [19].

Possion's ratio and Young's modulus are commonly used data for material properties. The values were assigned to the materials of each part of the model according to Table 1. Each docking unit was automatically identified as fully bound by Workbeach, and the contact surface was derived as a connecting surface.

According to the literature [20], the material properties of ligaments are shown in Table 2.

Ligaments were divided by T3D2 (Truss-3D-2node) unit, and the specific anatomical data and related material parameter settings are shown in Table 2. A facet joint capsule was added, and the facet joint was used as a contact model.

### 2.5. Validity Verification of Lumbar Three-Dimensional Finite Element Model

The effectiveness of thoracolumbar finite element model was verified regarding the stress and boundary constraints under normal physiological conditions of thoracolumbar. A torque load of 15 N·m was applied to a point on the upper surface of T12, and the bottom surface of T1 was fixed. The kinematic forces in six directions of forward bending, backward extension, left rotation, right rotation, left flexion, and right flexion were verified. The validation results were compared with those of Tencer A F to verify its validity [20].

### 2.6. Force Analysis of Finite Element Model

On the finite element model, the lower endplate of L_2_ cone was fixed, and two different forces were applied to simulate a variety of different stress states. The first method was applied perpendicular to the T12 cone surface 200 n, 400 n, and 600 n force of different motion state of stress changes. The second method was applying 16 Nm torque uniformly to each surface node of T_12_ under different conditions, such as forward bending, left- and right-side bending, extension, and torsion.

The model was loaded to obtain the displacement and stress of the model under different stress states.

The angular displacements of functional spinal unit (FSU) were measured as follows:

- A point *X* on the leading edge of T_12_ cone was taken, and the point was displaced to *X*_1_ after the vertical force was applied. The distance between two points was the displacement caused by the vertical force
- When the neutral position was taken, the two points *X* and *Y* on the front and rear edges of the T_12_ cone surface were connected to the two points *XY*. The cone was displaced to *X*_1_ and *Y*_1_ by the buckling or elongation moment, and the two points were connected to the two points *X*_1_*Y*_1_. The angle *β* between the two lines *XY* and *X*_1_*Y*_1_ was the rotation angle of the cone when it buckled or was subjected to the extensional moment
- The left and right points *X* and *Y* in the coronal position of T_12_ cone were taken, which were connected as line *XY*. The lateral bending or torsion torque was shifted to *X*_1_ and *Y*_1_, and the two points were connected as *X*_1_*Y*_1_. The angle *β* between the two lines *XY* and *X*_1_*Y*_1_ was the rotation angle of the cone under lateral bending or torsion moment

The average stiffness *K* of FSU are calculated:

(1) $$\begin{array}{c} K=\frac{F}{L},\\ K=\frac{F_{X}}{\beta }. \end{array}$$

In the above equations, *F* is the force on the cone, *L* is the displacement caused by the cone, *F_X_* is the moment when the cone is loaded, and *β* is the rotation angle when the moment is exerted. The unit is (Nm/degree) under compression (100 N/mm).

### 2.7. Establishment of a Three-Dimensional Finite Element Model of Minimally Invasive Fusion of Lumbar Spine and Its Force Analysis

DePuy spine model interbody fusion cage (Johnson & Johnson) was used, and the corresponding data was imported into ANSYS. The corresponding data is shown in Table 3. The fusion cage was inserted into the intervertebral space from the right oblique at 45° to the bottom surface. The specific construction method was that proposed in literature [20, 21]. The lower surface of L_5_ vertebral body was fixed, and a surface load of 400 N was applied uniformly perpendicular to the upper surface of L_3_ vertebral body, with an additional movement torque of 6 N·m. In ANSYS, the following operations were executed after loading of the model. (I) The spatial position coordinates of the anterior, posterior, and left and right four points on the L_4_-L_5_ surface were connected into lines, and the included angles between the lines represented the included angles between the upper surfaces of two adjacent vertebral bodies. The absolute value of the difference of the included angles before and after loading, *α*, was its angular displacement. (II) The angular displacement from L_3_ to L_4_ was recorded in the same way. (III) The stress change of each part was recorded.

### 2.8. Establishment of a 3D Finite Element Model of the Lumbar Pedicle Screw and Rod System

The UPASS2 pedicle screw rod system from WEGO, Shandong, was used. The interbody fusion cage was DePuy spine from Johnson & Johnson, and the corresponding data was imported into ANSYS. The intervertebral disc was divided into four zones on the front and back, and only annulus fibrosus, nucleus pulposus, and cartilage were retained in the first and forth zones. The fusion cage was inserted oblique from left to right into the L_4/5_ intervertebral space to assist bilateral pedicle screw rod fixation, and the point and direction of the Wiltsc approach was simulated. The specific construction method was that proposed in literature [22]. The lower surface of the S_1_ vertebral body was fixed, and a surface load of 500 N was applied uniformly perpendicular to the upper surface of the L_3_ vertebral body, with an additional movement torque of 10 N·m. In ANSYS, the following operations were executed after loading of the model. (I) The spatial position coordinates of the anterior, posterior, and left and right four points on the L_4_-L_5_ surface were connected into lines, and the included angles between the lines represented the included angles between the upper surfaces of two adjacent vertebral bodies. The absolute value of the difference of the included angles before and after loading, *α*, was its angular displacement. (II) The angular displacement from L_3_ to L_4_ was recorded in the same way. (III) The stress change of each part was recorded according to the software.

### 2.9. Statistical Methods

SPSS 19.0 was employed for data statistics and analysis. Mean ± standard deviation ($\overset{®}{x}$ ± s) was how measurement data were expressed, and percentage (%) was how count data were expressed. The pairwise comparison was performed by one factor analysis of variance. The difference was statistically considerable with *P* < 0.05.

## 3. Results

### 3.1. Comparison of the Efficacy of PVP and PKP

A total of 150 patients were analyzed. The height of the anterior edge and the middle of the wound cone after the operation in the two groups was remarkably higher than that before the operation (*P* < 0.05), and both were higher than those in the control group (*P* < 0.05). The PKP group had remarkably greater changes than the PVP group (*P* < 0.05, Figures 1 and 2). The postoperative kyphotic angle of the two groups was remarkably lower than that before the operation (*P* < 0.05), and the kyphotic angle of the two groups was smaller than that of the control group (*P* < 0.05), while the PKP group was more remarkably reduced than the PVP group (*P* < 0.05) (Figure 3). The postoperative VAS and ODI scores of the two groups were lower than those before the operation (*P* < 0.05), but there was no statistical difference between the two groups (*P* > 0.05), and both were higher than the control group (*P* < 0.05). Moreover, within 2 to 24 months after surgery, neither the VAS score nor the ODI score was statistically substantial (*P* > 0.05, Figures 4 and 5).

### 3.2. Establishment of 3D Finite Element Model of Cone

The human spine obtained by the CT scan is shown in Figure 6.

The CT image-based 3D finite element models are shown in Figures 7 and 8.

All the data was imported into ANSYS to generate the finite element model of the human spine T_12_-L_2_ according to the material parameters (Figure 9).

### 3.3. Force Analysis of Finite Element Model of Normal T_12_-L_2_ Segment

The source of force and boundary conditions on the spine were kept unchanged, and the magnitude of the force was changed to obtain the ultimate relationship between the displacement, stress, and force of the spine under different motion states. The details are shown in Figures 10 and 11.

From Figures 10 and 11, the vertebral body had the largest displacement when bending and flexing on the left side, and the stress was the largest when extending backward. Moreover, the changes in the spine force and the maximum displacement and the maximum stress basically conformed to the linear change law, which was also consistent with the linear elastic material of the model material of each part of the spine. These changes were consistent with clinical data.

The results of the lumbar finite element model in the three symbolic states of forward flexion, dextral flexion, and left flexion are analyzed in Figure 12; the two results were consistent with each other.

### 3.4. The Force Analysis of 3D Finite Element Model of the Lumbar Minimally Invasive Fusion System

The 3D finite element model of minimally invasive lumbar spine fusion was established by ANSYS, and the specific diagram is shown in Figure 13.

The force analysis of the finite element model was also carried out, and the angular displacement occurring in the L_4_~L_5_ section and the angular displacement occurring in the L_3_~L_4_ section are shown in Figure 14.

According to Figure 13, after the pedicle screw was added, the range of motion of the spine segment did not change remarkably, that is, the pedicle screw will not cause a substantial impact on the spine.

### 3.5. The Force Analysis of 3D Finite Element Model of the Lumbar Pedicle Screw and Rod System

The 3D finite element model of the lumbar pedicle screw and rod system was established by ANSYS. The specific diagram is shown in Figure 15.

The force analysis of the finite element model was performed, and the angular displacement and stress changes in the L_4/5_ section are shown in Figure 16.

## 4. Discussion

Due to the lack of methods and quantitative indicators for the accurate evaluation of thoracolumbar unstable fractures in elderly patients before and after surgery, the specific relationship between the damage degree and the mechanical harm is not clear, and the selection of treatment timing and methods is not accurate in clinical practice. Therefore, this research was developed to carry out in-depth mechanical studies for the elderly thoracolumbar unstable fractures before and after surgery, and fine analysis of the changes in the unstable fractures before and after surgery was implemented. It was hoped to provide scientific evidence to improve the above theory and improve the treatment effect.

In this research, 150 patients were studied, among which 75 patients in the surgery group were treated with PKP and 75 patients in the surgery group were treated with PVP. The results showed that the height of the anterior edge and the middle of the injured cone were remarkably higher after surgery than before surgery (*P* < 0.05), and the PKP group had greater changes than the PVP group (*P* < 0.05). At 2 to 24 months after surgery, the kyphosis of both groups was remarkably lower than that of the preoperative group (*P* < 0.05), and the decrease of PKP group was more substantial than that of PVP group (*P* < 0.05). VAS and ODI scores after surgery were lower than those before surgery (*P* <0.05), but there was no statistical difference between the two groups (*P* > 0.05). There was no statistical significance in VAS score and ODI score within 2 to 24 months after operation (*P* > 0.05), which indicated that both PVP and PKP can achieve satisfactory therapeutic effect, but PKP had a slightly better therapeutic effect than PVP. Zhang et al. (2017) [23] conducted an online meta-analysis of 32 studies involving 2,852 patients to compare the VAS score, ODI, kyphotic angle correction, and refracture occurrence. It was believed that both PKP and PVP performed well in treating OVCF. However, PKP had better pain relief and improved ODI score, while PVP had advantages in kyphotic angle and reduced fracture incidence. Chang et al. (2015) [24] concluded that PVP required less surgical time through a meta-analysis of prospective randomized trials. Moreover, compared with PKP, there was no substantial statistical difference in postoperative VAS and ODI scores, and PVP was still a safe and reliable treatment of first choice. This was basically consistent with the results of this research.

A finite element model (Th_12_L_2_) based on 3D images was constructed using CT digital imaging and medical communication in healthy controls or patients, and then motion pressure was simulated on the spinal model. For two spinal models, loads on the 12th thoracic vertebra (Th_12_) due to compression, flexion, extension, transverse bending, and axial rotation were examined in virtual space. Then, regarding the application of equivalent vertebrae stress, the 3D finite element analysis of the vertebral body was carried out to collect the movement state change data of the vertebral body under different stresses. Yan et al. (2016) [25] used aluminum-free glass polyacrylate cement (GPC) with an elastic modulus close to that of natural bone to establish a finite element model and analyzed it. It was found that GPC can produce low stiffness and stress in cancellous bone. The stress at the junction of the GPC and the cortical bone of the vertebral body was closer to the stress value of the natural vertebral body, so it showed good adaptability, mechanical, and biocompatibility. GPC is a material that may replace traditional polymethyl methacrylate cement to treat OVCF. The simulation results were compared with those obtained in this research, which proved the validity of the simulation results of this research.

After the effectiveness of the model was verified, the models of the minimally invasive intervertebral fusion system and the intervertebral pedicle screw rod system were established. In addition, the motion and stress analysis of the two were performed, and the effectiveness was verified. Compared with previous experiments, the validity of the two models was verified. After the collection of motion and stress data, it was concluded that the use of the two different internal fixation methods did not have a substantial effect on the movement of the vertebral body.

## 5. Conclusion

Both PVP and PKP can achieve satisfactory treatment results, and PKP had a slightly improved effect than PVP. Massive motion data of 3D finite element models of vertebral bodies were collected through verification experiments, and 3D finite element models of two different fixation methods of minimally invasive intervertebral fusion system and intervertebral pedicle screw rod system were established. Through the collection of the movement data of the two, it was proved that the two had no substantial effect on the normal intervertebral movement. Through this experiment, data proof and confirmatory experiments can provide data support for the selection of clinical treatment means and timing and provide ideas for the construction of new therapeutic instruments. However, only some basic data was collected, and the therapeutic effect was not analyzed, which has certain limitations for the choice of therapeutic means. However, with the development of new technologies and materials, there will be more choices of internal fixation and bone grafting for elderly thoracolumbar unstable fractures. In short, this experiment provides certain reference value for the validation of 3D finite element and biomechanical data of thoracolumbar vertebra.

## Figures and Tables

**Figure 1:** Comparison of the height of the front edge of the cone before and after the operation (∗*P* < 0.05 compared with that before operation; ^*P* < 0.05 compared with the control group; #*P* < 0.05 compared with PKP).

**Figure 2:** Comparison of the height of the injured vertebrae before and after the operation (∗*P* < 0.05 compared with that before operation; ^*P* < 0.05 compared with the control group; #*P* < 0.05 compared with PKP).

**Figure 3:** Comparison of kyphotic angle before and after surgery (∗*P* < 0.05 compared with that before operation; ^*P* < 0.05 compared with the control group; #*P* < 0.05 compared with PKP).

**Figure 4:** Comparison of VAS scores before and after surgery (∗*P* < 0.05 compared with that before operation; ^*P* < 0.05 compared with the control group; #*P* < 0.05 compared with PKP.)

**Figure 5:** Comparison of ODI scores before and after surgery (∗*P* < 0.05 compared with that before operation; ^*P* < 0.05 compared with the control group; #*P* < 0.05 compared with PKP).

**Figure 6:** CT imaging of the spine of a healthy male ((a) the coronal plane, (b) the cross section, and (c) the sagittal plane).

**Figure 7:** 3D finite element diagram of the spine (the enlarged part was the interosseous ligament model).

**Figure 8:** Schematic diagram of the intervertebral disc model.

**Figure 9:** T_12_-L_2_ segment finite element model.

**Figure 10:** The relationship between maximum displacement (DMX) and force (the dotted line represented the trend line of the maximum displacement under the three forces).

**Figure 11:** The relationship between stress maximum (SMX) and force (trend line of maximum stress under three kinds of stress).

**Figure 12:** Stress distribution of T_12_-L_2_ bone finite element model ((a) was the state of vertebral flexion; (a) was dextral vertebrae; (c) was left flexion of vertebrae).

**Figure 13:** Illustration of the 3D finite element model of the lumbar spine minimally invasive fusion.

**Figure 14:** The angular displacement of each segment of the model under different forces.

**Figure 15:** 3D finite element diagram of the pedicle screw rod system.

**Figure 16:** The maximum value of the range of motion and stress between the L_4/5_ segments of the model.

**Table 1:** Model material properties.

	Possion's ratio (*μ*)	Young's modulus (MPa)	Material model
Compact bone	0.3	12000	Anisotropy
Cancellous bone	0.2	100	Isotropy
Fiber ring	0.45	92	Isotropy
Nucleus pulposus	0.499	1.0	Viscoelasticity
Annulus matrix	0.51	3.36	Isotropy

**Table 2:** Material properties of ligaments.

	Density (ton/mm^3^)	Possion's ratio (*μ*)	Modulus of elasticity (MPa)	Cross-sectional area (mm^2^)	Unit number
Anterior longitudinal ligament	1.1 × 10^−9^	0.4	30	6.1	5
Posterior longitudinal ligament	1.1 × 10^−9^	0.4	20	5.4	5
Ligament flavum	1.1 × 10^−9^	0.4	10	50.1	3
Supraspinous ligament	1.1 × 10^−9^	0.4	1.5	13.1	2
Interspinous ligament	1.1 × 10^−9^	0.4	10	13.1	5
Capsular ligament	1.1 × 10^−9^	0.4	10	46.6	7
Intertransverse ligament	1.1 × 10^−9^	0.4	11	40	2

**Table 3:** Elements and nodes of finite element model of cone implant.

Site	Element type	Element number	Node number
Cortical bone	Three-dimensional	496,000	57,000
Cancellous bone	Three-dimensional	277,000	41,000
Screw system	Three-dimensional	128,000	30,000
Cage (rectangle)	Three-dimensional	21,000	4,700
Cage (cylindrical)	Three-dimensional	28,000	5,500

## Data Availability

The data used to support the findings of this study are included within the article.
